The article "Comparison of Proximate and Phytonutrient Compositions of Cashew Nuts and Apples from Different Geographical Areas of Burkina Faso" was published in 2022. Journal: Biomed Res Int.

# Comparison of Proximate and Phytonutrient Compositions of Cashew Nuts and Apples from Different Geographical Areas of Burkina Faso

**DOI:** 10.1155/2022/1800091

**Published:** 2022-10-11

**Authors:** Roger Dakuyo, Kiessoun Konaté, Abdoudramane Sanou, Kabakdé Kaboré, Hemayoro Sama, David Bazié, Mamounata Diao, Mamoudou Hama Dicko

**Affiliations:** ^1^Laboratory of Biochemistry, Biotechnology, Food Technology and Nutrition (LABIOTAN), Department of Biochemistry and Microbiology, University Joseph KI-ZERBO, 03 BP 7021 Ouagadougou, Burkina Faso; ^2^University of Dedougou, Burkina Faso; ^3^Laboratory of Biochemistry and Applied Chemistry (LABIOCA), Department of Biochemistry and Microbiology, University Joseph KI-ZERBO, 03 BP 7021 Ouagadougou, Burkina Faso

## Abstract

The cashew plant is an allogamous plant that produces two types of fruits: the nut and the cashew apple. The present study was conducted to perform a comparison of proximate and phytonutrient compositions of cashew (*Anacardium occidentale* L.) nuts and apples from different geographical areas of Burkina Faso. For this purpose, 60 samples of apples and kernels were collected from the three main cashew cultivation areas. The nutritional potential of cashew nuts and apples produced was evaluated to enhance their food processing. Protein, carbohydrates, lipids, dietary fibers, ascorbic acid, tannins, anthocyanins, chlorophyll, lycopene, and *β*-carotene contents were assessed. The results revealed high contents of lipids (50.42 ± 2.3 g/100 gDW), proteins (22.32 + −1.8 g/100 gDW), and starch (12.05 ± 1.27 g/100 g DW) in almonds. Apples, on the other hand, are rich in lipids, ascorbic acid (387.45 ± 17.4 mg/100 g), soluble sugars (387.45 ± 17.4 mg/100 g,), and pigments (lycopene, anthocyanin, *β*-carotene, and chlorophyll). In summary, almonds may be suitable as a source of lipids and related products. Apples can be used as natural antioxidants and produce juices. All of these data are important clues for cashew by-product processing. These results obtained provide a scientific basis for their food and economical valorization of cashew fruits.

## 1. Introduction

The cashew tree, *Anacardium occidentale* L., is a perennial crop that contributes to the socioeconomic development of several countries in the world [1]. It is cultivated in several countries of Africa (West and East), South America, and Asia (India, Vietnam, etc.). It is a plant that can reach more than 10 m of height depending on the climate and the nature of the soil. *Anacardium* plants are adapted to the humid tropical climate. World cashew nut production is estimated at 7 101 967 tons (FAOSTAT, 2021). Cashew nut production in Africa represents about 65% of the world's production, amounting to 4 666 351 tons (FAOSTAT, 2021). West Africa is the largest cashew-producing region worldwide, with 1 795000 tons of raw cashew nuts harvested in 2018, or 49% of the world supply. The cashew sector provides income to an estimated 10 million people in Africa [2]. In recent years, cashew has become the second largest export crop in West Africa by economic value, after cocoa [2]. Despite being the hub of global cashew production, just about40% of raw cashews are processed in West Africa, while 90% of production is processed in India and Vietnam [2]. In Burkina Faso, the cashew tree initially used to regenerate the plant cover has now become an important source of income for rural populations thanks to the technological, nutritional, and medicinal potential of its fruits. In 2020, it occupied 148,636 ha (FAOSTAT, 2021) for a production of 162 105 tons. The nuts of its fruits, in particular, constitute a real export commodity. Cashew nut exports were estimated at 117 billion XOF in 2018 [3] for 135 000 tons and represented the third largest agricultural export product after cotton and sesame. The main cashew nut-producing regions in Burkina Faso are the Cascades, the Centre-West, the Hauts-Bassins, and the South-West [4], which have an average rainfall between 650 and 1 200 mm/year (Fontès & Guinko, 1995). Currently, cashew cultivation is expanding with the increase of orchards. Burkina Faso, ranking 6th in Africa and 10th in the world, is one of the largest cashew producers in the world (FAOSTAT, 2021). Producers are interested in its cultivation because of its fruits, but also and especially its bark, leaves, and roots used in folk medicine [5]. The secondary metabolites present in *Anacardium* plants which display great antioxidant and antimicrobial effects [1].

The article "Comparison of Proximate and Phytonutrient Compositions of Cashew Nuts and Apples from Different Geographical Areas of Burkina Faso" was published in 2022. Journal: Biomed Res Int.

The cashew fruit comes in two parts: the nut, which is the true organic fruit, and the apple, which is called the false fruit. The cashew fruit is edible and used for therapeutic purposes making it both a food and medicinal plant (Oliveira et al., 2020). The juicy apple is consumed as food; but for conservation reasons and because of its astringent taste, which is not much appreciated by consumers, the apple is often abandoned on tree. Its moderate consumption is also explained by certain prejudices such as its incompatibility with milk. Indeed, it is reported that the consumption of apples with milk is fatal [6]. Although cashew apples are rich in polysaccharides [7], thousands of tons of cashew apples rot every year in the production orchards. As for the nut, it includes the shell, almond, and balsam; but it is especially the almond that is prized because it contains a lot of fat. The almond is used to make peanuts and sometimes as a substitute for milk powder in the manufacture of chocolate [8], while the shell is often used to produce energy by pyrolysis [9]. Studies in some regions have shown that apples and cashew almonds have high nutritional potential due to proteins [10], minerals, ascorbic acid, lycopene, carbohydrates, essential amino acids, etc. [11, 12]. The nectar of the cashew fruit has interesting antifungal (Oliveira et al., 2020) and antioxidant properties because of its richness in bioactive compounds [13, 14]. They also contain many types of pigments such as chlorophyll, anthocyanins, and carotenoids including beta-carotene, a provitamin A.

At the same time, the use of food by-products rich in bioactive compounds and which have an interesting nutritional value is developing today [15]. Embracing nutritional qualities, biological activities, and technological properties of plant byproducts in functional food formulation is actively studied [16]. Biological activities of respective components of the apple and cashew byproducts indicate important health promoting properties [17, 18]. Therefore, knowledge of the production area allowing to optimize the nutritional potential of the fruits is required that would allow to identify the favorable area for the establishment of orchards available for agroindustry. In short, this study will provide the scientific basis of these two by-products (nuts and apples) of cashew for better food and economic development.

## 2. Material and Methods

### 2.1. Plant Material

#### 2.1.1. Sample Collection

Cashew (*Anacardium occidentale* L.) fruits (Figure 1) were harvested from orchards in Burkina Faso during the 2019-2020 season. It is about cashew apple and cashew nut. The fruits were collected in the three largest producing regions of Burkina Faso, i.e., in the regions of Sud-Ouest at Gaoua (10° 17′ 57″ N, 3° 15′ 3″ W), Haut-Bassins, at Bobo-Dioulasso (11° 10′37.7″ N, 4° 17′ 52.4″ W), and Cascades, at Banfora (10° 37′ 60″ N, 4° 46′ 0″ W). In each orchard where samples were collected, a codification was made. This is consisted of dividing the plot into four subplots along the diagonals. From each subplot, 200 g of fresh apples and 500 g of cashew nuts were collected. The nuts were collected under the cashew trees where they sometimes stayed for up to 5 days depending on the orchard. The apples are picked directly from the plant or collected under the plant if they are firm. The apples were packed in coolers at 4 °C, to prevent their alteration and transported to the laboratory for analysis. The nuts were transported in fiber bags.

The article "Comparison of Proximate and Phytonutrient Compositions of Cashew Nuts and Apples from Different Geographical Areas of Burkina Faso" was published in 2022. Journal: Biomed Res Int.

For some analyses, fruits from neighboring production areas with similar growing conditions were included in the same sample and coded (Figure 2).

### 2.2. Production of Almond and Apple Flours

The nuts were crushed with manual pruning shear and then shelled. The almonds were obtained after a manual sorting operation. The almonds separated from the shells were dried in a controlled ventilated dryer (Prolab dryer) at 50 °C for 24 h and then dehulled. The dehulled kernels were oven dried at 65 °C for 24 h to reduce the humidity. The kernels were de-oiled in Soxhlet using n-hexane. The de-oiled almonds are oven dried for 2 hours at 50 °C to evaporate the hexane, and the obtained flours were used for assays. The apples were cut and dried in the sun (room temperature, about 30 °C) for 72 h and then in a ventilated dryer for 48 h at 40 °C. The dried apples were ground with a blender (MICROTRON®MB800), and the produced flour (Figure 3) was collected for analysis. The humidity of the flour obtained was 7 ± 2% for apples and almonds.

### 2.3. Assessment of Macronutrient Contents

Crude proteins were assessed by method described by [19] with slight modifications by [20]. Samples (500 mg) of apple and almond flours were homogenized in 10 mL of 0.1 M NaCl; the mixture was stirred (a150 rpm/min) for 5 h at 25 °C. The extract was collected after centrifugation at 4400 rpm for 30 min at 4 °C. 50 *μ*L of each extract was added 250 *μ*L of Bradford reagent. After incubation for 2 min, absorbances were read at 595 nm. A standard curve (*y* = 1.3138*x* + 0.0119; *R*^2^ = 0.999) was built using BSA as standard.

Total sugars were assessed by the phenol-sulfuric acid method [21] with few modifications. Absorbances were read on the spectrophotometer (EPOCH, BioTek Instruments Inc., USA) at 490 nm. Glucose was used as standard allowing to build a linear plot (*y* = 0.0107*x* + 0.9804; *R*^2^ = 0.998).

The total fat content of the samples was assessed by gravimetrical method according to the standard of AOAC 2003.05 (2012) using a Soxhlet apparatus (R040605, Gerhardt, Germany). Fat content is calculated using the following equation:

(1) $$\begin{array}{c} \text{Fat content}\left(\%\text{DM}\right)=\frac{\text{W}1-Wo}{Ws}\text{x}100, \end{array}$$

where *W*_0_ is the weight of the empty balloon (g), *W*_1_ is the weight of the flask after extraction and drying (g), and *W*_s_ is the initial sample weight (g).

Total carbohydrate content was assessed by subtracting the sum of protein, fat, and ash percentages (dry weight basis) of the sample from 100% [22].

Potential energy value was estimated using the Atwater coefficients. The calorific value of the sample is calculated [23] as follows:

(2) $$\begin{array}{c} \text{Energy value}=\text{P}\times 4\text{ Kcal}+\text{G}\times 4\text{ Kcal}+\text{L}\times 9\text{ Kcal}=\text{X}\frac{\text{kcal}}{100\text{g}}, \end{array}$$

where *P*, *G*, and *L* are the proportions of proteins, carbohydrates, and lipids, respectively.

The article "Comparison of Proximate and Phytonutrient Compositions of Cashew Nuts and Apples from Different Geographical Areas of Burkina Faso" was published in 2022. Journal: Biomed Res Int.

*Starch content* was assessed according to the spectrometric method described previously [24]. Rich starch was used as a standard, allowing to obtain a linear curve (*y* = 0.0549*x* − 0.0329; *R*^2^ = 0.9902).

*The dietary fiber* content was assessed using the gravimetric method **AOAC 991.43** with few modifications [25]. *α*-Amylase [*α*-1,4-D-glucan 4-glucanohydrolase, EC 3.2.1.1] from *Aspergillus orizae* and Amyloglucosidase [1,4-*α*-D-Glucan glucohydrolase, EC 3.2.1.3] from *Aspergillus niger* (lyophilized powder, 30-60 units/mg protein (biuret), ≤0.02% glucose) were used as digesting enzymes.

The water content was assessed by drying at 105 °C for 24 h in a steam room (NF V 03-707).

### 2.4. Assessment of Minerals and Ascorbic Acid Contents

Minerals such as zinc, iron, magnesium, manganese, potassium, calcium, sodium, and chlorine were quantified by atomic absorption spectroscopy (PerkinElmer, Waltham, MA), ICP- OES (inductively coupled plasma optical emission spectroscopy) (Varian Inc./Agilent Technologies), and ICP-MS (inductively coupled plasma mass spectroscopy) (Agilent Technologies). The method is based on that of Borowiak et al. [26]. The contents of the samples were assessed using a calibration curve (0-50 *μ*g) for each measured element. The levels are calculated by the following equation:

(3) $$\begin{array}{c} C1=\frac{\text{Co}*\text{V}}{Pe}\;C=\frac{\text{C}1*100}{\%\text{DM}}, \end{array}$$

where *C* = mineral content (concentration) in dry matter (mg/kg or ppm), *C*_1_ = mineral content in ash, *C*_0_ = standard mineral content, %*DM* = percentage in dry matter, *V* = dilution volume, and *Pe* = test sample.

*Ascorbic acid:* Ascorbic acid contents were assessed on the basis of the decolorization of *2,6*-dichlorophenolindophenol (DCPIP) by ascorbic acid [27] with slight modifications. 150 *μ*L of DCPIP (0.2 mM) was added to 50 *μ*L of an aliquot of the almond and apple extracts. The absorbances were read with a spectrophotometer at 515 nm against a blank consisting of 150 *μ*L of DCPIP and 50 *μ*L of distilled water. Values are extrapolated to a standard curve with ascorbic acid in the concentration range 10 *μ*g/mL to 100 *μ*g/mL (*y* = 0.0179*x* + 0.1781; *R*^2^ = 0.9918). Ascorbic acid contents are expressed as mg ascorbic acid equivalents per 100 g dry matter (mg EAA/100 g DM).

### 2.5. Assessment of Pigment Contents

*β*-Carotene, chlorophyll, and lycopene contents were assessed by adapting the methods described, respectively, by Wu et al. [28] and Kovalevskaya *et al.* [29]. Fresh apples and almonds (300 mg) were mixed with 3 ml of 95% ethanol. The mixture was kept for 10 min on ice and centrifuged for 1 min at 4500 rpm. For *β*-carotene and lycopene, the absorbances were read at different wavelengths, and the contents are calculated according to the following equations:

(4) $$\begin{array}{c} \text{Lycopene}\left(\frac{\text{mg}}{100\text{ml}}\right)=-0.0458\;{\text{A}}_{663}+0.372\;{\text{A}}_{505}–0.0806\;{\text{A}}_{453}, \end{array}$$

(5) $$\begin{array}{c} \beta -\text{carotene}\left(\frac{\text{mg}}{100\text{ml}}\right)=0.216\;{\text{A}}_{663}–0.304\;{\text{A}}_{505}+0.452\;{\text{A}}_{453}, \end{array}$$

(6) $$\begin{array}{c} \text{Total Chlorophyll}\left(\frac{\mu \text{g}}{\text{mL}}\right)=6.1\;{\text{A}}_{665}+20.04\;{\text{A}}_{649}, \end{array}$$

where the letter *A* with the numbers underscore were the absorbances of the supernatant.

The article "Comparison of Proximate and Phytonutrient Compositions of Cashew Nuts and Apples from Different Geographical Areas of Burkina Faso" was published in 2022. Journal: Biomed Res Int.

### 2.6. Assessment of Tannins, Anthocyanins, and Phytate Contents

The levels of hydrolysable tannins were quantified according to the method of [30] using tannic acid as standard. The results were expressed as mg tannic acid equivalent (GAE) per g dry extract (mgGAE/100 g). The hydrolysable tannins are determined by the following formula:

(7) $$\begin{array}{c} \text{Hydrolysable tannins}\left(\%\right)=\frac{\text{A}\times \text{Mw}\times \text{V}\times \text{DF}}{\varepsilon \lambda }\times \text{W}, \end{array}$$

where *A* is the absorbance, *Mw* is the molecular weight of tannic acid (1701.19 Da), *V* is the volume of extract used, *DF* is the dilution factor, *ε*_*λ*_ is the 2169 mol, and *W* is the sample weight (g).

Total phytate contents were assessed on a spectrophometric assay using phytic acid as standard [31]. The assay was performed with 2.0 mL of Wade reagent (0.03% (w/v) FeCl_3_ and 0.3% sulfosalicylic acid) and 3.0 mL of the eluted sample. The absorbances were read at 500 nm using spectrophotometer (EPOCH, BioTek Instruments Inc., USA).

Total anthocyanin contents (TAC) were assessed by the pH differential method AOAC (2005.02) with some modifications made by [32]. The absorbances were read with a spectrophotometer at two wavelengths (520 and 700 nm). The results were expressed as follows: cyanidin-3-o-sambubioside (C3SE) equivalents per liter, and the levels are obtained using the following formulas:

(8) $$\begin{array}{c} \text{A}=\left({\text{A}}_{520\text{nm}}-{\text{A}}_{700\text{nm}}\right)\text{pH }1.0-\left({\text{A}}_{520\text{nm}}-{\text{A}}_{700\text{nm}}\right)\text{pH }4.5, \end{array}$$

TAC is calculated as cyanidin-3-glucoside equivalents:

(9) $$\begin{array}{c} TAC\left(\frac{mg}{L}\right)=\frac{\text{A}*{\text{M}}_{w}*\text{DF}*1000}{\varepsilon }, \end{array}$$

where *A*: absorbance; *M*_W_: molecular weight of cyanidin-3-glucoside (449.2 g/mol); *DF*: dilution factor; and *ε*: molar extinction coefficient (26 900 mM^−1^ cm^−1^).

The article "Comparison of Proximate and Phytonutrient Compositions of Cashew Nuts and Apples from Different Geographical Areas of Burkina Faso" was published in 2022. Journal: Biomed Res Int.

### 2.7. Statistical Analysis

Graphs and calculations of the different concentrations were done using, Excel 2016, and XLSTAT 2016 was used for analyses of variance. Principal Component Analysis was performed using R software version 4.0.2 (2020).

## 3. Results and Discussion

### 3.1. Proximate Composition and Physicochemical Parameters

The two edible parts of the cashew fruit (*Anacardium occidentale* L.) showed totally different levels of moisture, protein, carbohydrates, fats, and total ash. Results reveal that although almonds and apples are all part of the cashew fruit, their biochemical compositions are very different (Table 1). Indeed, the water content varied between 7.99 ± 0.6 and 10.15 g/100 g FW for almonds and 83.64 ± 0.86 and 86.27 ± 0.78 for apples. These results clearly show that apples contain a significant amount of water, which explains their difficult conservation by producers compared to almonds and gives them a juicy appearance. Almonds and apples contain minerals on average 3.81 ± 0.33 g/100 g DW and 3.22 ± 0.4 g/100 g DW, respectively. The contents of the mineral fraction of both parts are close, but their composition is certainly different considering their nature.

Protein contents oscillated from 19.32 ± 3.4 and 23.14 ± 0.72 for almonds and 6.32 ± 0.92 and 7.15 ± 1.42 for apples. These data are similar to those of [4]. Cashew kernels are thus an important source of protein that can be used as ingredients for supplementary foods. Proteins are essential for the body's well-being because they perform structural and functional functions. Among specificities, studies have shown that almonds are rich in glutamic acid, arginine, aspartic acid, leucine, valine, and serine [10, 33]. Interestingly, leucine is an essential amino acid, so it must be provided to the human body. The consumption of cashew almonds would therefore be very beneficial and can cover some essential energy needs of the organism.

Almonds are very rich in fat (50.42 ± 2.3), while apples only contain traces (2.32 ± 0.54 g/100 gDW). These results are similar to those obtained by Rico et al. (48.3 ± 1.6 g/100 gDW), in a previous study on cashew kernels conducted in India [33]. The slight difference observed may be related not only to the influence of edaphic and environmental factors but also to the nature of used fertilizers [34]. Previous study reported similar fat contents of 13.8 g for 28 cashew kernels or 49.28 g/100 g [34]. This level of fat in cashew kernels confers potential uses in the process of butter, cheese, peanut, etc. Therefore, cashew kernels have comparable oilseed potential to other known oilseeds such as cotton seeds [35] but lower than peanuts and palm nuts [36]. Nevertheless, cashew almond oil is essential for human health because it is rich in unsaturated fatty acids (oleic and linoleic acid), vitamin E and proteins [37]. Almonds contained between 17.5 ± 2.5 and 21.12 ± 1.5 g/100 gDW of soluble sugars and 22.25 ± 2.4 and 25.52 ± 1.82 of total carbohydrates (Table 1). On a dry weight basis, the total carbohydrate content of cashew almonds is not negligible. It appeared that nearly 50% of its sugars are made up of starch, which gives the doughy or gelatinous aspect to the almond flour mixed with water. As for apples, they are very rich in total carbohydrates and reducing sugars. More than 85% of the dry weight of apples is made up of total carbohydrates, of which about 60% are soluble sugars. Cashew almonds contained dietary fiber in interesting proportions (12.05 ± 1.27 g/100 g DW). Levels of fibers found in this study are lower than those found by [38], who found levels of 16.04 g/100 g DW. The dietary fiber content also represents a significant proportion of the sugars present in almonds, which is very beneficial from a nutritional point of view [39]. In fact, dietary fiber helps reduce risk factors associated with the development of various chronic diseases, such as obesity, cardiovascular disease, and type 2 diabetes, by promoting the reduction of weight, blood sugar, and lipid profile [40]. Fibers are among the most used ingredients in functional foods, representing more than 50% of the total ingredients on the market [41]. They are also used as a food and pharmacological supplement [40]. Fruit fibers have an advantage over cereal fibers because they have a better water and oil retention capacity, more fermentable in the colon, and contain less phytic acid [42]. The energy value of almonds is quite high (566.45-645.21 Kcal/100 g of dry weight). This high fat content could explain the fact that almonds are classified as energy foods. Apples, although rich in carbohydrates, have presented lower energy values (279.75-396.82 Kcal/100 g of dry weight).

The article "Comparison of Proximate and Phytonutrient Compositions of Cashew Nuts and Apples from Different Geographical Areas of Burkina Faso" was published in 2022. Journal: Biomed Res Int.

### 3.2. Micronutrient Content

The trace elements quantified in this study are Mg, Cu, Mn, Fe, Zn, K, Na, Ca, P, and Cl (Figure 4). Both parts of the cashew fruits cultivated in Burkina Faso are very rich in potassium (K) with contents reaching 650 mg/100 g DW, a value higher than the average value (622 mg/100 g DW) found in other world regions [33]. After potassium, sodium (425 ± 15 mg/100 g), is the most abundant mineral in cashew almonds, followed by phosphorus (402.8 ± 17.24 mg/100 g), chlorine (386.2 ± 12.4 mg/100 g), magnesium (224.6 ± 14.1 mg/100 g), iron (47.8 ± 8.2 mg/100 g), and calcium (28.9 ± 5 mg/100 g). Cashew apples, in addition to potassium, contain some minerals in interesting quantities such as phosphorus (186.2 ± 12.4 mg/100 g), magnesium (146.6 ± 12.4 mg/100 g), iron (62.5 ± 5.2 mg/100 g), and sodium (54.8 ± 7.2 mg/100 g). Elements such as copper, zinc, and manganese were found in trace amounts in both almonds and apples. Present data are in agreement with those found by some previous works ([43]; Preethi *et al.,* 2021), with slight differences that can be explained by the methods used or by the nature of the soil. Levels of minerals in edible fruits are interesting because they are cofactors for certain proteins including metallo-enzymes and are involved in the formation of tissues and in certain hormonal biosynthesis [44].

### 3.3. Ascorbic Acid, Pigments, Phytates, and Tannins Content

Different parts of the plants in general are rich in various pigments that give them different colors [45]. For the cashew fruit, it is the apples that are very rich in various pigments (Table 2). The almonds, except for chlorophyll, contain very little pigment. Lycopenes are the most abundant pigments in apples (294.5 ± 24 mg/100 g), followed by anthocyanins (88.64 ± 11.5 g/100 g), *β*-carotenes (54.2 ± 8.94 mg/100 g), and chlorophyll (27.48 ± 6.45 mg/100 g). These pigments, in addition to giving the yellow-red or dark-orange color of apples, have important antioxidant properties. The results of this study are comparable with a study conducted in Venezuela on raw cashew apple juice, where lycopene and *β*-carotene contents of 580 ± 50.0 mg/100 g and 40 ± 6.2 mg/100 g, respectively, were found [46]. According to a recent study, lycopenes have enough interesting pharmacological properties as they prevent diabetes mellitus, cancer, liver disorders, and certain cardiac complications and can reduce the risk of diseases related to oxidative stress [47]. These data are similar to those found in a study of cashew apples in Brazil concerning *β*-carotene content [48]. *β*-Carotene is a provitamin A, nutritionally essential because it is metabolized to retinol (equivalent approximately 1/12), whose oxidation produces the retinal essential for the vision [28]. Health and nutrition interests on beta carotene consumption include immune system modulation, quenching singlet oxygen, free radical scavenging, improvement of gap-junction communication, induction of hepatic enzymes that detoxify carcinogens, and reduction of the risk of cardiovascular disease and cancer [49]. This study revealed that the levels of anthocyanins in cashews from Burkina Faso were largely higher than those found in Brazil [50]. This difference could be explained by different varieties of cashew trees which produce fruits of different phenotypes [4]. According to a study, pluviosity, edaphic, meteorological, and photoperiod conditions and biotic stresses could also affect the level of anthocyanins that regulate apple color [51]. Moreover, it is said that anthocyanins, which are antioxidant pigments, have attracted a lot of interest for their potential preventive and/or therapeutic effects on health, including prevention of obesity, cardiovascular diseases, antibacterial, anti-inflammatory, and anticancer effects [52]. Also, high level of anthocyanins was greatly correlated with the antioxidant activity of fruits (Legua et al., 2021).

The article "Comparison of Proximate and Phytonutrient Compositions of Cashew Nuts and Apples from Different Geographical Areas of Burkina Faso" was published in 2022. Journal: Biomed Res Int.

As for tannins and phytates, they are known for their anti-nutritional properties because of their complexation with macromolecules and minerals in the body, reducing their bioavailability [53]. Anti-nutritional factors are compounds that decrease the bioavailability of nutrients by interfering in their absorption. In this study, we quantified tannins and phytates. In addition, anti-nutritional factors present in fruit and oilseeds form complexes with proteins, divalent cations (iron, calcium, etc.), and digestive enzymes, reducing their bioavailability [54]. They are present in both compartments of *Anacardium occidentale* L. fruit. Tannins are more abundant in apple (204.8 ± 26.5 mg/100 g) than in almond (64.32 ± 12.4 mg/100 g), while phytates present higher levels in almond (89.34 ± 18.45 mg/100 g) compared to apples (41.72 ± 9.2 mg/100 g) (Table 2). Both hydrolysable (gallic and ellagic acid esters) and condensed (proanthocyanidins) tannins can form complexes with proteins and reduce their digestibility. They negatively impact the absorption of bivalent minerals (iron, copper, zinc, etc.) as well as the reserves of these micronutrients [55]. It is therefore may not be advisable for pregnant women and children to consume large quantities of foods rich in tannins [56]. Fortunately, hydrolysable tannins can be degraded in apples by enzymatic and thermal treatments [57]. In addition, at low doses, tannins may be interesting in human health because of their antioxidant activity and inhibition of the growth of various groups of microorganisms such as fungi, yeasts, viruses, and bacteria [58]. Moreover, consumption of foods containing low concentrations of tannins has also been reported to contribute to the reduction of high blood pressure and serum lipid constituents (King-Thom *et al.,* 1998). Phytic acid is also known to reduce the absorption of certain minerals such as bivalent cations (copper, zinc, iron, etc.) [59, 60].

The article "Comparison of Proximate and Phytonutrient Compositions of Cashew Nuts and Apples from Different Geographical Areas of Burkina Faso" was published in 2022. Journal: Biomed Res Int.

Cashew apples are very rich in ascorbic acid (387.45 ± 17.4 mg/100 g) in contrast to almonds which contain only traces of it (18.13 ± 6.2 g/100 g DW) (Table 2). The results differ significantly according to collection area; this is explained by the fact that all three sample collection sites are in the same climatic zone with very little soil variation. The differences between the compound contents of the different types could be explained by the cashew varieties grown in the collection area.

These values are similar to those found in cashew apples from Brazil, displaying ascorbic acid contents of 279.37 mg. 100 g^−1^ [50]. Another study in Ghana on cashew apple juice found average ascorbic acid contents of 231.4 mg. 10 mL^−1^ [61]. However, Assunção and Mercadante [48] showed lower levels of ascorbic acid (121.65 ± 8.06 mg/100 mL). This difference may be attributable to the extraction method used in this study as a continuous extraction cycle was used and that could certainly explain the high levels of ascorbic acid in our cashew apple extracts. Thus, cashew apples are an important source of ascorbic acid. Indeed, they contain more ascorbic acid than oranges, which are known to be rich in this molecule (13 mg/L of juice) [62, 63]. Ascorbic acid is particularly important for strengthening of the immune system involved in the renewal and functioning of certain white blood cells [64], collagen biosynthesis, etc. Consumption of cashew apples would be an alternative to the increasing demand for ascorbic acid, especially for low-income populations. In synergy with vitamin E, beta-carotene, selenium, zinc, and other minerals, ascorbic acid is able to trap the excess of free radicals present in the body, which accelerate cellular aging [65]. As such, it contributes to the prevention of cardiovascular diseases, certain cancers, cataracts, and neurodegenerative diseases [66]. Ascorbic acid is recognized as a powerful antioxidant that helps strengthen the immune system. At the beginning of the COVID-19 pandemic, foods rich in ascorbic acid were highly recommended to cope with the SARS-CoV-2 coronavirus [67].

## 4. Conclusion

The analysis of the proximate composition and phytonutrient contents of cashew apples and almonds from the three localities under climate conditions of Burkina Faso revealed a difference among samples. Such difference was much governed by their intrinsic differences rather than their geographical origin. It was confirmed that cashew apples are good sources of carbohydrates, ascorbic acid, and pigments (lycopene, anthocyanin, *β*-carotene, and chlorophyll), while almonds have great levels of fat, protein, and various minerals. These results suggest that cashew apples and almonds can be valorized in the manufacturing industry, particularly in the functional food and cosmetic industries. These studied by-products can be a source of additional income, especially for rural populations. Presented findings may provide a basis for potential product formulations including apple and cashew almonds products.

The article "Comparison of Proximate and Phytonutrient Compositions of Cashew Nuts and Apples from Different Geographical Areas of Burkina Faso" was published in 2022. Journal: Biomed Res Int.

## Figures and Tables

**Figure 1:** Parts of the cashew fruit (apple and nut).

**Figure 2:** Codification of the sample. CK: Cascades kernels; HK: Hauts-Bassins kernels; SK: South-West kernels; CA: Cascades apples; HA: Hauts-Bassins apples; SA: South-West apples.

**Figure 3:** Different steps in the production of flour samples prior to analysis.

**Figure 4:** Mineral content. For the needs of graphic representation, the concentrations of Cu, Mn, and Zn have been multiplied by 10 (∗10); CK: Cascade kernel; SK: South-West kernel; HK: Haut-Bassins kernel; CA: Cascade apples, SA: South-West apples; HA: Haut-Bassins apples.

**Table 1:** Proximate composition and potential energy values of cashew kernels and apples.

Sample	Humidity	Proteins	Fats	Soluble sugars	Dietary fibers	Starch	Total carbohydrates	Ashes	Energy value
	*(g/*100 *g FW)*	*(g/*100 *g DW)*	*(g/*100 *g DW)*	*(g/*100 *g DW)*	*(g/*100 *g DW)*	*(g/*100 *g DW)*	*(g/*100 *g DW)*	*(g/*100 *g DW)*	*(kcal/*100 *gDW)*
*Cashew kernels*									
CK_1_	10.15 ± 0.5^a^	22.15 ± 0.8^a^	51.15 ± 4.42^a^	17.5 ± 2.5^ab^	3.85 ± 1.01^a^	11.5 ± 1.02^ab^	22.25 ± 2.4^a^	4.45 ± 0.21^a^	566.45
CK_2_	8.96 ± 0.45^a^	21.31 ± 1.2^a^	50.03 ± 2.78^a^	19.54 ± 2.21^ab^	4.10 ± 0.75^a^	12.63 ± 0.9^a^	24.72 ± 3.15^a^	3.94 ± 0.15^a^	613.67
CK_3_	9.35 ± 0.62^a^	23.14 ± 0.72^a^	49.35 ± 5.14^a^	19.01 ± 1.84^ab^	3.65 ± 0.89^a^	10.5 ± 0.65^b^	23.39 ± 1.97^a^	4.12 ± 0.62^a^	612.75
SK_1_	7.99 ± 0.6^a^	21.87 ± 1.4^a^	48.98 ± 3.13^a^	19.68 ± 0.87^ab^	4.04 ± 1.21^a^	9.84 ± 1.12^b^	25.51 ± 2.04^a^	3.64 ± 1.02^a^	607.02
SK_2_	8.65 ± 0.32^a^	22.03 ± 2.2^a^	49.12 ± 4.00^a^	19.45 ± 1.21^ab^	5.21 ± 1.13^a^	10.51 ± 0.72^b^	24.98 ± 1.7^a^	3.87 ± 0.75^a^	608.00
SK_3_	8.86 ± 0.75^a^	21.15 ± 3.32^a^	48.36 ± 1.94^a^	21.12 ± 1.5^a^	4.85 ± 0.61^a^	8.23 ± 0.23^c^	25.52 ± 1.82^a^	3.97 ± 1.01^a^	604.32
HK_1_	9.05 ± 0.8^a^	19.86 ± 1.84^a^	53.21 ± 3.05^a^	20.78 ± 2.15^a^	4.35 ± 1.01^a^	12.54 ± .85^a^	23.69 ± 1.45^a^	3.24 ± 0.75^a^	641.45
HK_2_	8.32 ± 0.27^a^	20.10 ± 2.71^a^	54.25 ± 2.72^a^	19.14 ± 1.75^ab^	3.62 ± 1.5^a^	11.4 ± 1.62^ab^	22.6 ± 2.41^a^	3.05 ± 0.65^a^	645.21
HK_3_	8.74 ± 0.4^a^	19.32 ± 3.45^a^	52.45 ± 4.50^a^	20.27 ± 1.63^a^	4.15 ± 1.34^a^	13.61 ± 2.14^a^	24.22 ± 1.5^a^	4.01 ± 0.62^a^	630.41

*Cashew apples*									
CA_1_	85.15 ± 1.24^a^	5.96 ± 0.23^a^	2.64 ± 0.08^a^	60.72 ± 3.24^a^	11.52 ± 1.54^a^	LQ	88.23 ± 1.32^a^	3.17 ± 0.52^a^	286.48
CA_2_	83.75 ± 0.87^a^	5.65 ± 0.95^a^	2.43 ± 0.10^ab^	62.12 ± 1.97^a^	10.25 ± 2.02^b^	LQ	88.88 ± 2.41^a^	3.05 ± 0.75^a^	288.95
CA_3_	84.25 ± 1.5^a^	5.07 ± 0.8^a^	3.52 ± 0.07^a^	62.45 ± 2.26^a^	13.26 ± 1.6^a^	LQ	88.6 ± 1.15^a^	2.81 ± 1.10^a^	297.76
SA_1_	86.27 ± 0.78^a^	5.51 ± 1.02^b^	2.15 ± 0.14^ab^	61.3 ± 2.13^a^	9.92 ± 0.55^b^	LQ	88.13 ± 1.2^a^	3.21 ± 0.84^a^	282.59
SA_2_	84.44 ± 0.92^a^	7.15 ± 1.42^a^	1.63 ± 0.21*b*^b^	60.12 ± 3.12^a^	12.25 ± 0.8^ab^	LQ	87.88 ± 1.05^a^	3.34 ± 0.52^a^	279.75
SA_3_	84.23 ± 1.02^a^	6.32 ± 0.92^a^	2.55 ± 0.16^ab^	62.03 ± 4.45^a^	11.75 ± 2.4^ab^	LQ	88.21 ± 1.32^a^	3.01 ± 0.75^a^	283.35
HA_1_	85.62 ± 1.15^a^	6.78 ± 1.75^a^	3.10 ± 0.20^a^	59.45 ± 2.44^a^	13.05 ± 1.75^a^	LQ	86.17 ± 2.04^a^	3.95 ± 1.23^a^	396.82
HA_2_	83.64 ± 0.86^a^	6.95 ± 1.3^a^	3.02 ± 1.45^a^	61.75 ± 3.54^a^	13.52 ± 0.97^a^	LQ	86.79 ± 1.63^a^	3.24 ± 0.78^a^	297.98
HA_3_	86.15 ± 0.79^a^	7.12 ± 1.4^a^	2.95 ± 0.90^a^	63.62 ± 5.12^a^	12.92 ± 1.32^a^	LQ	86.15 ± 0.94^a^	3.78 ± 0.25^a^	305.51

CK: Cascade kernel; SK: South-West kernel; HK: Haut-Bassins kernel; CA: Cascade apples; SA: South-West apples; HA: Haut-Bassins apples. LQ: limit of quantification. Under score numbers 1, 2, and 3 indicate the three groups of samples by region.

The article "Comparison of Proximate and Phytonutrient Compositions of Cashew Nuts and Apples from Different Geographical Areas of Burkina Faso" was published in 2022. Journal: Biomed Res Int.

**Table 2:** Pigment and anti-nutritional factors content.

Samples	*β*-Carotene	Lycopene	Chlorophyll	Anthocyanins	Phytates	Tannin	Ascorbic acid
	*(mg/*100 *gDW)*	*(mg/*100 *gDW)*	*(mg/*100 *gDW)*	*(mg/100 gDW)*	*(mgPAE/*1*00 gDW)*	*(mgGAE/*1*00 gDW)*	*(mgAAE/*1*00 gDW)*
*Cashew kernels*							
CK_1_	LQ	LQ	0.45 ± 0.12^a^	LQ	92.45 ± 10.26^a^	55.00 ± 4.57^ab^	12.20 ± 1.10^c^
CK_2_	LQ	LQ	0.20 ± 0.07^b^	LQ	111.89 ± 7.45^a^	42, 4 ± 3.87^ab^	11.98 ± 0.93^c^
CK_3_	LQ	LQ	0.38 ± 0.24^a^	LQ	118.63 ± 6.31^a^	35 ± 5.14^ab^	21.78 ± 0.95^b^
SK_1_	LQ	LQ	0.12 ± 0.06^b^	LQ	95.41 ± 5.21^a^	108.12 ± 8.44^a^	14.04 ± 1.21^bc^
SK_2_	LQ	LQ	0.24 ± 0.11^ab^	LQ	75.48 ± 7.15^ab^	93.10 ± 7.15^a^	10.72 ± 0.78^c^
SK_3_	LQ	LQ	0.17 ± 0.04^b^	LQ	87.15 ± 7.82^a^	64.65 ± 5.23^ab^	31.13 ± 3.65^a^
HK_1_	LQ	LQ	0.27 ± 0.13^ab^	LQ	49.48 ± 5.24^b^	35.21 ± 3.32^b^	20.75 ± 2.97^b^
HK_2_	LQ	LQ	0.39 ± 0.22^a^	LQ	58.75 ± 7.6^b^	38.12 ± 8.45^ab^	31.12 ± 4.34^a^
HK_3_	LQ	LQ	0.25 ± 0.07^ab^	LQ	87.63 ± 9.58^a^	28.95 ± 7.48^b^	25.81 ± 2.42^a^

*Cashew apples*							
CA_1_	63.25 ± 5.12^ab^	348.15 ± 19.23^a^	17.9 ± 3.45^b^	102.24 ± 9.15^a^	55.35 ± 5.15^a^	145.14 ± 2.56^b^	278.45 ± 15.25^a^
CA_2_	65.15 ± 4.17^ab^	284.12 ± 25.45^ab^	22.5 ± 4.19^b^	110.51 ± 11.15^a^	62.21 ± 4.21^a^	135.25 ± 4.18^b^	312.51 ± 12.51^a^
CA_3_	31.31 ± 4.62^b^	272.52 ± 22.75^a^	20.6 ± 2.15^b^	98.56 ± 7.94^a^	32.15 ± 4.86^b^	139.45 ± 4.25^b^	302.98 ± 22.10^a^
SA_1_	82.01 ± 7.58^a^	198.74 ± 32.25^b^	32.18 ± 7.94^ab^	101.64 ± 12.23^a^	25.15 ± 3.45^b^	240.5 ± 4.15^a^	225.40 ± 13.45^a^
SA_2_	38.32 ± 4.15^b^	323.15 ± 19.21^a^	28.45 ± 5.62^ab^	82.15 ± 7.45^b^	46.32 ± 4.15^a^	234.64 ± 6.5^a^	250.32 ± 10.56^a^
SA_3_	42.25 ± 10.28^b^	304.25 ± 21.2^ab^	19.24 ± 2.74^b^	94.69 ± 6.12^ab^	29.78 ± 3.56^b^	133.25 ± 6.2^b^	245.12 ± 14.13^a^
HA_1_	58.56 ± 2.15^ab^	215.54 ± 12.62^a^	31.24 ± 4.25^ab^	75.81 ± 14.15^b^	43.94 ± 5.54^a^	262.62 ± 7.26^a^	285.78 ± 18.16^a^
HA_2_	61.85 ± 5.22^b^	272.05 ± 24.26^ab^	42.15 ± 8.12^a^	84.67 ± 11.32^b^	61.62 ± 6.43^a^	140.18 ± 8.51^b^	294.15 ± 16.15^a^
HA_3_	29.25 ± 2.84^b^	321.45 ± 16.94^a^	29.45 ± 6.34^ab^	69.46 ± 9.21^b^	25.24 ± 4.85^b^	224.32 ± 11.36^a^	289.54 ± 9.75^a^

CK: Cascade kernel; SK: South-West kernel; HK: Haut-Bassins kernel; CA: Cascade apples; SA: South-West apples; HA: Haut-Bassins apples; PAE: phytic acid equivalent; TAE: tannic acid equivalent; AAE: ascorbic acid equivalent; LQ: limit of quantification. Under score numbers 1, 2, and 3 indicate the three groups of samples by region.

The article "Comparison of Proximate and Phytonutrient Compositions of Cashew Nuts and Apples from Different Geographical Areas of Burkina Faso" was published in 2022. Journal: Biomed Res Int.

## Data Availability

The data used to support the findings of this study are available from the corresponding author upon request.
